# A Meta-Analysis of Incidence of Catheter-Related Bloodstream Infection with Midline Catheters and Peripherally Inserted Central Catheters

**DOI:** 10.1155/2022/6383777

**Published:** 2022-03-12

**Authors:** Xin Chen, Min Liang

**Affiliations:** ^1^Department of Intensive Care Unit, Hangzhou Tumor Hospital Affiliated to School of Medicine, Zhejiang University, Hangzhou 310002, China; ^2^Department of Intensive Care Unit, Xiasha Campus, Sir Run Run Shaw Hospital Affiliated to School of Medicine, Zhejiang University, Hangzhou 310019, China

## Abstract

In order to provide reference for the prevention and treatment of CRBSI during clinical intravenous infusion therapy, this paper investigates the incidence of catheter-related bloodstream infection (CRBSI) in the treatment of midline catheters (MCs) and peripherally inserted central catheters (PICCs) by intravenous infusion. Web of Science, PubMed, Scopus, Embase, Cochrane Library, and ProQuest are searched to collect CRBSI-related studies on MC and PICC. The retrieval time is from the database construction to August 2020. Two researchers independently searched and screened literature quality evaluation and extracted data according to inclusion and exclusion criteria, and RevMan 5.3 software was used for analysis. Eleven studies are included, with a total of 33809 patients. The incidence of CRBSI in the MC group is 0.599% (43/7079), and that in the PICC group is 0.4993% (133/26630). Meta-analysis showed that the incidence of CRBSI in the MC group is higher than that in the PICC group (OR = 0.72, 95% CI = 0.43–1.08, *P*=0.11), and the difference is statistically significant when low-quality studies are excluded (OR = 0.60, 95% CI = 0.39–0.93, *P*=0.02). There is no significant difference in the incidence of CRBSI between MC group and PICC group (*P* > 0.05), American subgroup (OR = 0.52), and British subgroup (OR = 4.86), the results of the two groups are opposite, and the incidence of CRBSI between the MC group and PICC group is statistically significant. There is no significant difference in the incidence of CRBSI between the adult and other subgroups (all *P* > 0.05). There is no significant difference in the incidence of CRBSI between the MC group and the PICC group (*P* > 0.05). Overall, the inter-study stability is general, the quality is good and the medium is good, and there is no obvious publication bias. The risk of CRBSI in MC and PICC is systematically evaluated and meta-analyzed for the first time. The incidence of CRBSI in MC group is lower than that in PICC group during intravenous infusion therapy. Under the same conditions, MC patients can be given priority for intravenous infusion therapy. More high-quality and child-related studies are needed to further evaluate and explore the risk of CRBSI between MC and PICC.

## 1. Introduction

Catheter-related bloodstream infection (CRBSI) is a serious complication of intravenous fluid therapy, which is closely related to the length of hospital stay, cost, and prognosis of patients [1]. CRBSI is defined as bacteremia or mycoemia with fever within 48 hours of catheter insertion or catheter removal (>38). Infection such as chills or hypotension and infection with no other clear source of infection other than vascular catheter infection are excluded [2]. Laboratory microbiology tests showed positive bacteria or fungi from peripheral venous blood cultures or pathogens of the same species with the same drug sensitivity results from catheter segments and peripheral blood cultures [2]. CRBSI is also the most common cause of hospital bacteremia, with treatment costs ranging from $32,000 to $69,332 [3–5].

Different infusion methods and tools lead to different incidence of CRBSI. Medium-length catheter is also called midline catheter (MC), the catheter length is 20–30 cm, and the catheter is inserted into the important vein, cephalic vein, or brachial vein from the upper arm through conventional puncture of the upper and lower fingers at the elbow fossa or ultrasound-guided technology. The tip of the catheter is located in the thoracic segment of the axillary vein or may reach the subclavian vein [6, 7]. The 2015 standard of nursing practice for intravenous infusion therapy of Infusion Nurses Society (INS) recommends that all drugs and fluids that can pass through peripheral superficial venous devices be used for medium-length catheters [8]. Medium-length catheter has the advantages of simple operation and fewer vascular complications, protecting blood vessels and reducing the pain of repeated puncture [8]. The incidence of CRBSI of MC is 0–0.9% [9, 10]. Peripherally inserted central catheter (PICC) is a catheter inserted through a peripheral vein, such as the arm vein or saphenous vein, with the tip reaching the superior vena cava or right atrium. PICC may be used for long-term chemotherapy drugs and prolonged antimicrobial therapy, total parenteral nutrition, or infusion of drugs unsuitable for peripheral intravenous administration [11, 12]. The incidence of CRBSI of PICC ranged from 0.3% to 7.3% [13–15].

Due to the low attention paid to MC studies in the early stage and the increasing number of studies in recent years, there is no systematic evaluation of the incidence of CRBSI in MC and PICC intravenous infusion therapy. Through systematic review and meta-analysis, this study explored the difference in the incidence of CRBSI between MC and PICC intravenous infusion therapies, in order to provide reference for the prevention and treatment of CRBSI during clinical intravenous infusion therapy.

## 2. Our Proposed Method

### 2.1. Search Strategy

Our research is carried out according to Preferred Reporting Item for Systematic Reviews and Meta-Analyses (PRISMA) eporting guidelines [16]: Computer search Web of Science, PubMed, Scopus, Embase, Cochrane Library, and ProQuest. Mesh term and synonyms are used for retrieval. Search terms are as follows: (1) midline catheter^*∗*^, midline venous catheter^*∗*^, midline peripheral cathe-ter^*∗*^, medium-term intravenous access^*∗*^; (2) PE-ripherally inserted central catheter∗, percutaneous indwelling central catheter^*∗*^, peripherally inserted central Catheter^*∗*^, PICC line^*∗*^, PICC^*∗*^; (3) Bacteremia, bacteriemia, septicemia, sepsis, infection^*∗*^. The retrieval time is from the database construction to August 2020.

### 2.2. Inclusion and Exclusion Criteria

Inclusion criteria were as follows. (1) Study type: experimental or observational studies related to CRBSI between MC and PICC. (2) Subjects: an observational study on the complications of CRBSI in patients receiving intravenous infusion therapy with MC or PICC and an experimental study on the intervention of MC and PICC on the complications of CRBSI in intravenous therapy. Exclusion criteria were as follows: (1) case report, review, comment, etc.; (2) non-human research literature; (3) secondary study; (4) <10 subjects; (5) repeated publications and other suspected duplicate reports; and (6) the report data are incomplete and relevant data cannot be obtained. Two researchers searched independently, first browsing the titles and abstracts and then reading the full text to determine the inclusion and exclusion of literature. In case of disagreement, they reached an agreement with a third-party researcher.

### 2.3. Literature Quality Evaluation

Since there are experimental and observational studies in the included studies, two researchers independently used the literature quality evaluation checklist proposed by Downs and Black [17] to evaluate the quality of the literature. Inventory evaluation includes 5 dimensions including report, external validity, internal validity, bias, and statistical analysis, with 27 items totaling 32 points. The quality of literature is divided into four levels according to the scores: excellent (≥26 points), good (20–25 points), medium (15–19 points), and poor (≤14 points).

### 2.4. Literature Screening and Data Extraction

The data are extracted using the template provided by the Cochrane Collaboration [18]. Two researchers independently extracted the data and checked them by a third researcher to establish a database. The data extraction content includes the first author and publication time of the literature, research method, research country, research time, research population characteristics, the number of MC and PICC, and the number of CRBSI occurrences.

### 2.5. Statistical Analysis

RevMan 5.3 software is used for meta-analysis. The count data used the odds ratio (OR) as the effect indicator, and the measurement data used the standard mean deviation (SMD) as the effect indicator. Each effect size is given its point estimate and 95% confidence interval (CI). The *I*^2^ statistic is used to assess heterogeneity [19]. If *I*^2^ > 50%, random effect model is used [20]. Subgroup or sensitivity analyses are performed for studies with significant heterogeneity, or descriptive analyses are performed only. Sensitivity analysis is performed by culling to check whether the statistical results had changed significantly. *χ*^2^ test is used for comparison between groups, and *P* ≤ 0.05 is considered statistically significant. A *P* value <0.05 is taken to indicate statistical significance. Publication bias is detected by funnel plot, and the greater the asymmetry, the greater the degree of bias.

## 3. Result

### 3.1. Literature Search Results

A total of 617 literatures are obtained through preliminary retrieval, and 11 literatures are finally included after preliminary screening by reading titles and abstracts and reading the full text. The literature screening process and results are shown in Figure 1.

### 3.2. Characteristics of Included Studies

Eleven articles are included, including 1 from China, 4 from the United States, 3 from the United Kingdom, and 1 each from Australia, Canada, and the Czech Republic. Two papers are abstracts of the conference. A total of 33,803 patients are included, including 7248 in the MC group and 26,714 in the PICC group, as shown in Table 1.

### 3.3. Risk of Bias Analysis

Among the 11 articles, 5 are good quality, 5 are medium quality, and 1 is poor quality.  Table 2 shows quality evaluation result of included literature.

### 3.4. Outcomes

Meta-analysis of 33809 patients in 11 studies shows that the incidence of CRBSI is 0.599% (43/7179) in the MC group and 0.499% (133/26630) in the PICC group. Heterogeneity among the studies is low (*I*^2^ = 40%), and the incidence of CRBSI in the MC group is lower than that in the PICC group by using the fixed effect model, with no statistical significance (OR = 0.72, 95% CI (0.48, 1.08), *P*=0.11). One study with poor quality [Sargent 1997] is excluded, and the heterogeneity among the studies is significantly reduced (*I*^2^ = 0). Using the fixed effect model, meta-analysis showed that the incidence of CRBSI in the MC group is lower than that in the PICC group, and the difference is statistically significant (OR = 0.60, 95% CI (0.39, 0.93), *P*=0.02).  Figure 2 presents result of incidence risk of CRBSI in the MC group and PICC group.  Figure 3 displays result for good and moderate quality research of incidence risk of CRBSI in the MC group and PICC group.

According to the different source countries of the research objects, the research is divided into the United States, the United Kingdom, and other country subgroups, of which for the United States subgroup, there is no heterogeneity among the studies (*I*^2^ = 0). Meta-analysis showed that the incidence of CRBSI in the MC group is lower than that in the PICC group, and the difference is statistically significant (OR = 0.52, 95% CI (0.31, 0.89), *P*=0.02). There is no heterogeneity among the studies in the British subgroup (*I*^2^ = 0). Meta-analysis showed that the incidence of CRBSI in the MC group is higher than that in the PICC group, and the difference is statistically significant (OR = 4.86, 95% CI (1.13, 20.96), *P*=0.03). Meta-analysis of subgroups in other countries showed that the incidence of CRBSI in the MC group is not statistically different from that in the PICC group (OR = 0.70, 95% CI (0.28, 1.78), *P*=0.45).  Figure 4 illustrates the result of each country subgroup of incidence risk of CRBSI in the MC group and PICC group.

According to the age of the research subjects, the research is divided into adult research and other subgroups. Other subgroups include children, adults, and studies that did not report the age of the research subjects. Among them, there is no heterogeneity among the adult subgroups (*I*^2^ = 0). Meta-analysis showed that the incidence of CRBSI in the MC group is not statistically different from that in the PICC group (OR = 0.64, 95% CI (0.27, 1.49), *P*=0.30); there is moderate heterogeneity between studies in other subgroups (*I*^2^ = 70%), suggesting that the heterogeneity between studies is large. Meta-analysis shows that the incidence of CRBSI in the MC group is not statistically different from that in the PICC group (OR = 1.52, 95% CI (0.26, 8.92), *P*=0.64).  Figure 5 shows the result of each age subgroup of incidence risk of CRBSI in the MC group and PICC group.

According to different research types, the research is divided into randomized controlled study (RCT) subgroups and retrospective cohort study (RC) subgroups, in which RCT subgroup meta-analysis showed that the incidence of CRBSI in the MC group is lower than that in the PICC group, and the difference is statistically significant (OR = 0.30, 95% CI (0.012, 7.69), *P*=0.47). There is low heterogeneity among the studies in the RC subgroup (*I*^2^ = 46%). Meta-analysis showed that the incidence of CRBSI in the MC group is not statistically different from that in the PICC group (OR = 0.73, 95% CI (0.48, 1.10), *P*=0.13).  Figure 6 presents the result of different study design subgroups of incidence risk of CRBSI in the MC group and PICC group.

### 3.5. Sensitivity Analysis

The 11 included studies are eliminated one by one. The sensitivity analysis showed that after arbitrarily excluding one of the studies, the combined OR = 0.63, 95% CI 0.43–93, which is similar to the total combined effect value, suggesting that the research results are stable and credible. Among the studies of good quality and medium quality, each study is eliminated one by one, and the results of the study did not change significantly.

### 3.6. Publication Bias

In the publication bias test, the funnel graph has good symmetry, and it can be considered that there is no obvious publication bias. Some studies are at the bottom of the funnel chart, suggesting that some studies are of poor quality.  Figure 7 shows funnel plots of incidence risk of CRBSI due to MC and PICC.

## 4. Clinical Analysis

The complication of intravenous infusion CRBSI is a serious complication, which prolongs the hospitalization time of patients, increases the cost of hospitalization, and even threatens the life safety of patients. Different infusion tools cause different incidences of CRBSI. PICC is a long-term use of central venous infusion access tool. After years of practice, clinical treatment techniques have become more and more perfect, but the high CRBSI caused by it is a problem that cannot be ignored. MC is a newly emerging intravenous infusion therapy tool in recent years, and it has been widely used in clinical practice. Both MC and PICC can develop CRBSI to varying degrees in intravenous infusion, but the risk of CRBSI is different. Many previous studies still have different opinions on the risk of CRBSI between MC and PICC. This study adopted a comprehensive search, a systematic review, and a meta-analysis method. We explored the risk of CRBSI between MC and PICC in order to provide a basis for the selection of appropriate infusion tools for subsequent intravenous infusion treatment.

The results of this study showed that the incidence of CRBSI in the MC group is lower than that in the PICC group, but the difference is not statistically significant (*P*=0.11). After excluding poor-quality studies, the results of meta-analysis showed that the incidence of CRBSI in the MC group is lower than that in the PICC group, and the difference is statistically significant (*P*=0.02). However, between the good-quality and medium-quality studies, the study results did not change after excluding each study, suggesting that the study concluded that the incidence of CRBSI in the MC group is lower than that in the PICC group. It is stable, reliable, and consistent with the conclusions of related studies.

In the subgroup analysis, the conclusion of the study from the United States is consistent with the final conclusion, confirming that the incidence of CRBSI in the MC group is lower than that in the PICC group. The articles are of poor quality, and 2 articles are of medium quality. Meta-analysis of adult study subgroups showed that the incidence of CRBSI in the MC group is not statistically different from that in the PICC group (*P*=0.30), and literature or poor-quality literature is eliminated one by one. The conclusions of the study did not change. Among them, 3 studies did not report the age of the study subjects. Whether it has an effect on the adult study subgroup is still unknown, suggesting the importance of complete data reporting in later studies. There is only one child study evaluating CRBSI risk in the MC group and PICC group. However, the quality of this study is moderate, and CRBSI did not occur in both groups. There is no reference for the CRBSI risk evaluation of children using MC and PICC, which suggests that later changes are needed.

## 5. Conclusion

In summary, the incidence of CRBSI in the MC group is lower than that in the PICC group during intravenous infusion therapy. Under the same conditions, MC can be considered as a priority for intravenous infusion therapy. In the future, more high-quality exploration of the risk of CRBSI between MC and PICC is still needed, and children's studies are needed to further evaluate the risk of CRBSI between MC and PICC.

The limitations of this article are as follows. (1) The overall research quality of the included studies is low, and there are few high-quality studies. (2) There is a possibility that some studies have not been retrieved. The included studies are all published Chinese and English documents, and the literature may be incomplete. (3) There is a certain statistical heterogeneity among the studies. Nevertheless, this study is still the first in this field to systematically evaluate and meta-analyze the risk of CRBSI between MC and PICC.

## Figures and Tables

**Figure 1:** Literature screening process and result of meta-analysis.

**Figure 2:** Result of incidence risk of CRBSI in the MC group and PICC group.

**Figure 3:** Result for good and moderate quality research of incidence risk of CRBSI in the MC group and PICC group.

**Figure 4:** Result of each country subgroup of incidence risk of CRBSI in the MC group and PICC group.

**Figure 5:** Result of each age subgroup of incidence risk of CRBSI in the MC group and PICC group.

**Figure 6:** Result of different study design subgroups of incidence risk of CRBSI in the MC group and PICC group.

**Figure 7:** Funnel plots of incidence risk of CRBSI due to MC and PICC.

**Table 1:** Basic characteristics of included literature.

Study, year	Country	Researching spells	Population	Design	MC (CRBSI/total)	PICC (CRBSI/total)
Tao, 2019	China	August 2016–September 2018	42–75 years old	RC	3/279	6/208
Seo, 2020	USA	November 2017–July 2018	≥18 years old	RC	0/82	1/50
Xu, 2016	USA	January 2015–May 2015	19–98 years old	RC	0/200	2/206
Caparas, 2014	USA	NR	Vancomycin is used for ≥6 days	RCT	0/30	1/28
Moureau, 2002	USA	April 1999–September 2000	1–101 years old	RC	14/5423	11/25707
Snooks, 2019	England	June 2017–December 2018	NR	RC	2/43	0/22
Barr 2012	England	January 1, 2001–May 31, 2011	≥18 years old	RC	12/648	0/43
Sargent, 1997	England	1995–1996	HIV sufferers	RC	7/12	2/18
Sharp, 2014	Australia	2004–2010	18–47 years	RC	0/231	0/97
Benali, 2013	Canada	NR	≤18 years old and ≥3 kg	RCT	0/69	0/84
Lisova, 2015	Czech	2013	23–90 years old	RC	5/162	4/167

RC: retrospective cohort; RCT: randomized controlled trial; NR: not reported.

**Table 2:** Quality evaluation result of included literature.

Study, year	Reporting	External validity	Bias	Confounding	Power	Total score	Grade
Sargent, 1997	4	3	3	2	1	13	Poor
Moureau, 2002	7	2	4	3	3	19	Moderate
Barr, 2012	9	3	3	3	2	20	Good
Benali, 2013	7	3	4	4	2	20	Good
Caparas, 2014	9	3	4	5	2	23	Good
Sharp, 2014	9	3	4	3	3	22	Good
Lisova, 2015	5	3	4	2	2	16	Moderate
Xu, 2016	10	3	4	4	2	23	Good
Snooks, 2019	5	2	3	3	2	15	Moderate
Tao, 2019	9	3	3	3	2	20	Good
Seo, 2020	9	3	5	2	1	20	Good

## Data Availability

The data used to support the findings of this study are available from the corresponding author upon request.
